The article "ZNF655 Promotes the Progression of Glioma Through Transcriptional Regulation of AURKA" was retracted in 2023. Reasons: unreliable results or conclusions; concerns about the data.

# ZNF655 Promotes the Progression of Glioma Through Transcriptional Regulation of AURKA

**DOI:** 10.3389/fonc.2022.770013

**Published:** 2022-02-24

**Authors:** Xu Chen, Chao Liu, Zhenyu Zhang, Meng Wang, Shewei Guo, Tianhao Li, Hongwei Sun, Peng Zhang

**Affiliations:** ^1^ Department of Neurosurgery, Tongji Hospital, Tongji Medical College, Huazhong University of Science and Technology, Wuhan City, China; ^2^ Department of Neurosurgery of the First Affiliated Hospital of Zhengzhou University, Zhengzhou City, China

**Keywords:** ZNF655, glioma, prognosis, phenotype, tumorigenesis, AURKA

## Abstract

**Objectives:**

Glioma has a high degree of malignancy, strong invasiveness, and poor prognosis, which is always a serious threat to human health. Previous studies have reported that C2H2 zinc finger (ZNF) protein is involved in the progression of various cancers. In this study, the clinical significance, biological behavior, and molecule mechanism of ZNF655 in glioma were explored.

**Methods:**

The expression of ZNF655 in glioma and its correlation with prognosis were analyzed through public datasets and immunohistochemical (IHC) staining. The shRNA-mediated ZNF655 knockdown was used to explore the effects of ZNF655 alteration on the phenotypes and tumorigenesis of human glioma cell lines. Chromatin immunoprecipitation (ChIP)-qPCR and luciferase reporter assays were performed to determine the potential mechanism of ZNF655 regulating Aurora kinase A (AURKA).

**Results:**

ZNF655 was abundantly expressed in glioma tissue and cell lines SHG-44 and U251. Knockdown of suppressed the progression of glioma cells, which was characterized by reduced proliferation, enhanced apoptosis, cycle repression in G2, inhibition of migration, and weakened tumorigenesis. Mechanistically, transcription factor ZNF655 activated the expression of AURKA by directly binding to the promoter of AURKA. In addition, downregulation of AURKA partially reversed the promoting effects of overexpression of ZNF655 on glioma cells.

**Conclusions:**

ZNF655 promoted the progression of glioma by binding to the promoter of AURKA, which may be a promising target for molecular therapy.

## Introduction

Glioma is the most common tumor of the human central nervous system, which is characterized by complex heterogeneity, high degree of malignancy, strong invasiveness, and poor prognosis (1, 2). In addition, gliomas are mainly composed of several subtypes, such as astrocytoma, oligodendroglioma, ependymoma, and neuroglioma hybrids (3, 4). Clinically, gliomas are usually classified into grades I to grade IV according to the degree of malignancy (5). Currently, traditional therapies include a combination of surgery, radiation, and chemotherapy (6, 7). Despite improved treatment outcomes in glioma patients, the median survival time is still only 12–18 months (8). In general, the solution of glioma as a challenging disease requires continuous exploration in the field of molecular biology to determine effective molecular therapy targets.

The article "ZNF655 Promotes the Progression of Glioma Through Transcriptional Regulation of AURKA" was retracted in 2023. Reasons: unreliable results or conclusions; concerns about the data.

Zinc finger proteins (ZFPs) are one of the most abundant proteins in eukaryotic genomes. Their functions are very diverse, including DNA recognition, RNA packaging, transcriptional activation, apoptosis regulation, protein folding and assembly, and lipid binding (9). Cys2His2 (C2H2)-type ZFPs have been widely explored, which could specifically identify the target sites in chromosomes and effectively regulate the expression of its target genes (10). Accumulating evidence reported that the abnormal expression of C2H2-type ZFPs participated in the progression of various tumors, including colorectal cancer, prostate cancer, and lung cancer (11–14). During recent years, specific transcription factors, especially C2H2-type ZFPs, have emerged as promising anticancer drug targets. Thalidomide is a promising anticancer drug that targets transcription factors and acts by inactivating ZFPs, which has been used as a treatment for hematological malignancies (15, 16).

Zinc-finger protein 655 (ZNF655), also known as Vav-interacting Kruppel-like protein-1 (Vik-1), belongs to the C2H2-type ZFP (17). This protein is involved in a variety of biological functions, such as embryonic development, cell differentiation, and hematopoiesis (18). In addition, a previous study clarified that ZNF655 was downregulated in glioma-associated endothelial cells, whose overexpression could inhibit the angiogenesis of glioma-associated endothelial cells (19). Moreover, ZNF655 possessed a promoting effect in the progression of non-small cell lung cancer (20). However, the biological functions and underlying molecular mechanisms of ZNF655 in glioma cells are still unknown. Therefore, the limited information of ZNF655 encouraged us to further analyze its potential role in gliomas.

This study was the first to identify the expression of ZNF655 in glioma samples and its association with prognosis through public datasets and immunohistochemical staining. Moreover, we performed *in vitro* and *in vivo* experiments to evaluate the effects of ZNF655 in glioma cells. The downstream target of ZNF655 was determined by human GeneChip and Ingenuity Pathway Analysis.

## Materials and Methods

### Immunohistochemical Staining

This study was approved by the Research Ethics Committee of the First Affiliated Hospital of Zhengzhou University. Human survival glioma tissue array (Outdo Biotech Company, Shanghai) included glioma tissue (n = 125; low grade, n = 49, high grade, n = 76) and normal tissue (n = 31), which was performed with immunohistochemical (IHC) staining to determine ZNF655 expression levels. Notably, the subtypes of glioma tissue included astrocytoma, oligodendroglioma, and glioblastoma. In brief, the tissues were successively immersed in xylene and alcohol for dewaxing and rehydration, repaired with sodium citrate buffer. After that, the tissues and primary antibodies (**Table S1**) were co-incubated at room temperature for 2 h, followed by the addition of a secondary antibody for 2 h. Subsequently, the tissues were stained with DAB and hematoxylin in turn. The total scores of immunohistochemical staining therewith were determined by staining percentage scores (classified as 1 (1%–24%), 2 (25%–49%), 3 (50%–74%), 4 (75%–100%)) and staining intensity scores (scored as 0: signal less color, 1: brown, 2: light yellow, 3: dark brown) and observed with a microscope.

The article "ZNF655 Promotes the Progression of Glioma Through Transcriptional Regulation of AURKA" was retracted in 2023. Reasons: unreliable results or conclusions; concerns about the data.

### Cell Culture

Human brain normal glial cells HEB and human glioma cells U87, U251, and SHG-44 were purchased from the Cell Bank of the Chinese Academy of Sciences (Shanghai, China), and the atmosphere was maintained at 37°C with 5% CO_2_. In addition, these cells were cultured in DMEM (Corning, Cat. No. 10-013-CVR) supplemented with 10% fetal bovine serum (FBS) (Ausbian, Cat. No. A11-102) and puromycin (Gibco, Cat. No. A11138-003).

### Target RNA Interferes With the Preparation of Lentiviral Vector

First, RNA interference (RNAi) against ZNF655 (shZNF655) or AURKA (shAURKA) and corresponding negative control (shCtrl) were designed (**Table S2**) and synthesized.

These sequences were ligated to BR-V-108 lentivirus vectors (Shanghai Bioscienceres, Co., Ltd., Shanghai, China) that carried the green fluorescent protein (GFP), respectively. The recombinant lentivirus vector plasmid was co-transfected into 293T cells with auxiliary plasmids (Helper 1.0, Helper 2.0). At the same time, the overexpressed sequence of ZNF655 (ZNF655) was constructed and inserted into the lentiviral vector BR-V-108. The NC group was used as corresponding negative control. After that, these lentiviruses were respectively infected with SHG-44 and U251 and cultured for 72 h. The GFP of the cells was observed under the fluorescence microscope (Olympus) to estimate the infection efficiency.

### Quantitative PCR

The RNA from SHG-44 and U251 cells was obtained with TRIzol reagent (Sigma, Cat. No. T9424-100m) and then reverse-transcribed into cDNA by HiScript Q RT SuperMix (Vazyme, Nanjing, China, Cat. No. R123-01), respectively. Subsequently, the mixed reaction solution composed of cDNA, corresponding primers (**Table S3**), and SYBR Premix (Vazyme, Nanjing, China) was performed to quantitative PCR (qPCR). The relative mRNA expression of ZNF655 was quantified with cycle threshold (Ct) values and normalized using the 2^–∆∆Cq^ method (21).

The article "ZNF655 Promotes the Progression of Glioma Through Transcriptional Regulation of AURKA" was retracted in 2023. Reasons: unreliable results or conclusions; concerns about the data.

### Western Blotting Analysis

SHG-44 and U251 cells were lysed, and the protein quality was detected by BCA Protein Detection Kit (HyClone-Pierce, South Logan, USA). The 10-µg protein was separated by SDS-PAGE (Invitrogen, Carlsbad, CA, USA), transferred to the PVDF membrane, and sealed with TBST solution. Afterward, the proteins with the primary antibody (**Table S1**) were incubated at 37°C for 2 h, and then with the secondary antibody at 4°C overnight. Finally, Millipore Immobilon Western Chemiluminescent HRP Substrate Kit (Millipore, Cat. No. RPN2232, Bedford, MA, USA) was used for color rendering and Chemiluminescent imager (GE, Cat. No. AI600, Chicago, IL, USA) observation.

### MTT Assay

The SHG-44 and U251 cells were inoculated at a density of 1,000/well on a 6-well plate for 14 days and then washed with phosphate buffer. After that, the cells were fixed with 4% paraformaldehyde (Sigma, Cat. No. P6148, St. Louis, MO, USA) of 1 ml for 60 min, stained with 500 μl Giemsa (Tripod Biotechnology, Cat. No. KGA229) for 20 min, washed, and dried with ddH_2_O. After that, the OD490 value was observed under a microplate reader (BioTek ELx800) for five consecutive days at the same time.

### Celigo Cell Counting Assay

The SHG-44 and U251 cells were cultured in a 96-well plate with a density of 2,000 cells per well. After that, the cells were counted by Celigo (Nexcelom, Lawrence, MA, USA) every day for 5 days. Accordingly, the cell proliferation curve was drawn by counting the number of GFP cells in each scanning orifice plate.

### Apoptosis Detection Assay

The SHG-44 and U251 cells were continuously cultured in 6-well plates for 7 days and then centrifuged. The cell precipitates were washed by precooled D-Hanks (pH = 7.2~7.4) and 1× buffer solution in turn. After resuspension, cells were precipitated and stained with Annexin V-APC (eBioscience, Cat. No. 88-8007-74) for 10–15 min; the apoptosis rate was analyzed and calculated by flow cytometry (Millipore, Cat. No. IX73).

### Cell Cycle Detection Assay

The SHG-44 and U251 cells were continuously cultured in 6-well plates for 7 days and then centrifuged. The cell precipitates were washed with PBS (pH = 7.2~7.4), precooled at 4°C and then fixed with 70% ethanol for at least 1 h. After that, the cells were centrifuged again to remove the fixed liquid. The cell precipitates were stained with 1.5 ml staining solution (40 × PI mother liquor (2 mg/ml): 100 × RNase mother solution (10 mg/ml): 1 × PBS = 25:10:1,000). Finally, the cell cycle distribution was detected by flow cytometry with a pass rate of 200–350 cells/s.

The article "ZNF655 Promotes the Progression of Glioma Through Transcriptional Regulation of AURKA" was retracted in 2023. Reasons: unreliable results or conclusions; concerns about the data.

### Wound-Healing Assay

The SHG-44 and U251 cells were cultured in the 96-well plate with a density of 5 × 10^4^ cells/well. The following day, the low concentration of serum medium was replaced, and the scratches were formed by nudging upward at the center of the 96-well plate with a scratch meter. After 0, 8, 24, and 30 h of cell migration, the width of the scratch area in the image was measured and the difference in cell migration ability was measured.

### Transwell Assay

The SHG-44 and U251 cells with a density of 5 × 10^4^ cells/well were incubated in the well-hydrated chamber (3422 Corning, Tewksbury, MA, USA). The inner chamber contained 100 μl of serum-free medium, and the external chamber contained 600 μl 30% FBS. The cell suspension was diluted with serum-free medium and then added to each chamber for a 24-h cultivation. After fixing with 4% formaldehyde, the migrating cells were stained with Giemsa. Finally, the cells were observed under the fluorescence microscope and photographed to estimate the migration capacity.

### Mouse Xenograft Model

All procedures involving mice and experimental protocols were approved by the Institutional Animal Care and Use Committees of the Neurosurgery, Tongji Hospital, Tongji Medical College, Huazhong University of Science and Technology. The 200-μl SHG-44 cells (about 4 × 10^6^ cells) with (shZNF655) or without (shCtrl) knockdown of ZNF655 were subcutaneously injected into 4-week-old female BALB/c nude mice (Beijing Viton Lihua, Beijing, China), which were divided into two groups (shCtrl, n = 5 and shZNF655, n = 5) for mouse xenograft models. The cells were subcutaneously injected into mice, and cultured animals were monitored for tumor growth in real time. On Day 9, the tumor was visible to the naked eye. Subsequently, data were collected once or twice every other week (weighing animals and measuring the length and diameter of tumors) until 65 days. Meanwhile, *in vivo* imaging (Berthold Technologies, Bad Wildbad, Germany) was performed to observe the tumor formation. On the 65th day, mice were sacrificed by cervical vertebrae and the tumors were weighed using electronic balance. Finally, the tumor tissues were removed from mice and incubated with antibody Ki67 (**Table S1**) for IHC staining.

### Human Apoptotic Antibody Array

The concentrations of 43 human apoptotic markers in the U251 cells were measured simultaneously using human apoptosis antibody array-membrane (Abcam, Cat. No. ab134001, Cambridge, MA, USA). After the cell protein was obtained, the product instructions were followed to detect the differential expression of the groups of shCtrl and shZNF655.

The article "ZNF655 Promotes the Progression of Glioma Through Transcriptional Regulation of AURKA" was retracted in 2023. Reasons: unreliable results or conclusions; concerns about the data.

### Affymetrix Human GeneChip PrimeView

Affymetrix Human GeneChip PrimeView combined with Affymetrix Scanner 3000 was performed to elaborate the molecular mechanism. Accordingly, the volcano plot and hierarchical clustering of the shCtrl and shZNF655 in U251 cells were presented by the differentially expressed genes (DEGs) with criterion of |Fold Change| ≥ 2 and false discovery rate (FDR) < 0.05. Furthermore, the significant enrichment of DEGs in the canonical pathway, and diseases or functions were investigated based on Ingenuity Pathway Analysis (IPA).

### Promoter Reporters and Dual-Luciferase Assay

The AURKA promoter region (chr20:56367390-56394196) was amplified, and the obtained fragment was cloned into the luciferase reporter vector GL002 (Promega, Madison, USA). Subsequently, U251 cells were transfected with 100 ng recombinant plasmid GL002-AURKA using 0.2 μl Lipofectamine 3000 Reagent (Thermo Fisher Scientific, Cat. No. L3000008, USA) and culture for 48 h. According to the Promega Dual-Luciferase system (Cat. No. E2940, Madison, USA) instructions, Firefly luciferase value and Renilla luciferase signals were determined.

### Chromatin Immunoprecipitation-qPCR Assay

According to the method provided in the literature to carry out the experimental operation (22), U251 cells were cross-linked with formaldehyde, lysed in SDS buffer, and sheared mechanically by sonication to fragment the DNA. Protein–DNA complexes were precipitated with 2 μg control rabbit IgG (CST, Cat. No. 2729), anti-Histone H3 (D2B12) XP^®^ Rabbit mAb (CST, Cat. No. 4620), and anti-ZNF655 (Novus, Cat. No. NBP1-78732, Littleton, CO, USA) antibodies, respectively. The complex was eluted from the antibodies, and the eluted DNA fragment was assessed by qPCR. Real-time PCR was performed using primers specific for the AURKA promoter (chr20:56367390-56394196) and SYBR premix (Vazyme). The AURKA primers are listed as follows: forward primer 5′-AGAACGTTCACTCGCCAGGTA-3′, reverse primer 5′-GCATCTGTGTTCTAGCCTTTCCA-3′.

### Statistical Analysis

Statistical analyses were accomplished by SPSS 19.0 with GraphPad Prism 8.0 software, and data were presented as the mean ± standard deviation. The independent Student’s t test was used to analyze the statistical significance between different groups, and p < 0.05 was considered statistically significant.

## Results

### High Expression of ZNF655 Predicts Poor Prognosis in Glioma Patients

We first analyzed the mRNA level of ZNF655 in human glioma (n = 518) and normal tissue (n = 207) from the public available database GEPIA2 (http://gepia2.cancer-pku.cn/#analysis). As shown in **Figure 1A**, the ZNF655 mRNA level was elevated in tumor tissues compared with the adjacent normal tissues. According to the database (http://gepia2.cancer-pku.cn/#survival), we further found that ZNF655 expression was positively correlated with overall survival (**Figure 1B**). Moreover, the results based on the Cancer Genome Atlas (TCGA) database further showed that the expression level of ZNF655 in glioblastoma (n = 155) was significantly higher than that of normal tissues (n = 5) (**Figure 1C**). The relationship between the expression level of ZNF655 and the survival time of glioblastoma was analyzed using the Kaplan–Meier method, finding that there was no significant correlation between them (**Figure 1D**). Subsequently, the expression of ZNF655 in glioma tissue (n = 125; low grade, n = 49, high grade, n = 76) and normal tissue (n = 31) was analyzed through IHC staining. The proportion of ZNF655-positive cells in glioma tissues was significantly higher than that in normal tissues (**Figure 1E**), as the quantitative results show in **Figure 1F**. According to the results of the IHC score, those higher than the median were defined as high expression of ZNF655, otherwise low expression. The high expression of ZNF655 in high-grade glioma tissues (47.4%) was significantly higher than that in normal tissues (0) (**Table 1**). Furthermore, the relationship between ZNF655 expression and tumor characteristics in patients with high-grade glioma was analyzed through Mann–Whitney (**Table 2**) and Spearman correlation coefficient (**Table 3**). Consistently, the mRNA expression of ZNF655 was elevated in glioma cell lines (U87, U251, and SHG-44) compared to human brain normal glial cells HEB (**Figure 1G**). These results together revealed that the expression of ZNF655 was positively correlated with the grade of glioma. Taken together, the high expression of ZNF655 may play an important role in glioma.

The article "ZNF655 Promotes the Progression of Glioma Through Transcriptional Regulation of AURKA" was retracted in 2023. Reasons: unreliable results or conclusions; concerns about the data.

**Figure 1:** Correlation analysis of the expression level of ZNF655 in glioma and its prognosis. **(A)** The mRNA level of ZNF655 in human glioma (n = 518) and normal tissue (n = 207) were analyzed from the public available database GEPIA2. **(B)** The relationship between high or low expression of ZNF655 and prognosis of glioma were analyzed in the GEPIA2 database. **(C, D)** Based on the TCGA database, the expression level of ZNF655 in glioblastoma and its correlation with survival were analyzed. **(E, F)** The expression of ZNF655 in glioma tissue (n = 125; low grade, n = 49, high grade, n = 76) and normal tissue (n = 31) were analyzed through IHC staining (×200 magnification and ×400 magnification), and quantitative results of ZNF655 in gliomas were shown. **(G)** The mRNA expression of ZNF655 was elevated in glioma cell lines (U87, U251, and SHG-44) and human brain normal glial cells HEB. **(H, I)** The mRNA and protein expression levels of ZNF655 in SHG-44 and U251 cells transfected with shRNA lentivirus were detected. The data were expressed as mean ± SD (n ≥ 3), **p < 0.01, ***p < 0.001.

**Table 1:** Expression patterns in glioma tissues and normal tissues revealed in immunohistochemistry analysis.

ZNF655 expression	High-grade glioma tissue		Normal tissue		p value
	Cases	Percentage	Cases	Percentage	
Low	40	52.6%	31	100%	<0.001
High	36	47.4%	0	–	

**Table 2:** Relationship between ZNF655 expression and tumor characteristics in patients with high-grade glioma.

Features	No. of patients	ZNF655 expression		p value
		Low	High	
All patients	76	40	36	
Age	76	40	36	0.200
Gender				0.123
Male	53	31	22	
Female	23	9	14	
Tumor size	75	39	36	0.634
Grade				0.013
III	28	20	8	
IV	48	20	28	

**Table 3:** Relationship between ZNF655 expression and tumor characteristics in patients with high-grade glioma.

		ZNF655
Grade	Spearman correlation coefficient	0.288
	Significance (two tails)	0.012
	N	76

### Knockdown of ZNF655 Suppresses the Progression of Glioma *In Vitro*

To assess the effects of ZNF655 in glioma, the shRNA-mediated knockdown of ZNF655 in SHG-44 and U251 cell lines was established. As illustrated in **Figure S1A**, more than 80% of GFP-labeled cells were observed, indicating successful cell infection. Furthermore, the consistent downregulation of ZNF655 at RNA (**Figure 1H**) and protein (**Figure 1I**) levels indicated its knockdown success in SHG-44 and U251 cells. shCtrl was the BR-V-108 vector with scrambled sequence for cell infection and as negative control; shZNF655 was the cell with downregulation of ZNF655. Therefore, SHG-44 and U251 cells were used to investigate the effect of altered ZNF655 expression on the phenotype of glioma cells. We continued to monitor cell viability for 5 days and found that the OD490 value of the shZNF655 group was significantly lower than that of the shCtrl group (p < 0.001) (**Figure 2A**). The results revealed that downregulation of ZNF655 weakened the proliferation of the SHG-44 and U251 cells. Based on the flow cytometry results, we found that the apoptosis ability of the shZNF655 group was significantly higher than that of the shCtrl group (p < 0.001) (**Figure 2B**). Furthermore, the effect of ZNF655 knockdown on the apoptosis signaling pathway in U251 cells was preliminarily investigated by human apoptotic antibody array. These findings indicated that knockdown of ZNF655 resulted in downregulation of Bcl-2, Bcl-w, clAP-2, IGF-I, IGF-II, sTNF-R1, sTNF-R2, and TNF-β (p < 0.05) (**Figure S1B**). Moreover, the proportion of the cell cycle in the G2 phase was sharply increased in the shZNF655 group compared with the control group, indicating that ZNF655 knockdown can arrest the cell cycle in G2 (**Figure 2C**). Additionally, the comparison of the scratch distance between the shZNF655 group and the shCtrl group during 30 h showed that the downregulation of ZNF655 led to the weakening of cell migration ability (p < 0.001) (**Figure 2D**). Consistently, the number of migratory cells in the shZNF655 group was obviously less than that in the shCtrl group under a microscope (p < 0.001) (**Figure 2E**). Western blotting (WB) results indicated that knockdown of ZNF655 in U251 cells decreased Akt phosphorylation, and downregulation of CDK1, CDK6, CCND1, and PIK3CA (**Figure S1C**). Collectively, the downregulation of ZNF655 suppressed glioma cell progression by reducing proliferation, enhancing apoptosis, disrupting the cycle, and impeding migration *in vitro*.

The article "ZNF655 Promotes the Progression of Glioma Through Transcriptional Regulation of AURKA" was retracted in 2023. Reasons: unreliable results or conclusions; concerns about the data.

**Figure 2:** The regulation effects of ZNF655 on cell proliferation, apoptosis, and migration in glioma cells. **(A)** MTT assay was performed to detect the cell proliferation rate of SHG-44 and U251 cells infected with shCtrl or shZNF655. **(B, C)** Flow cytometry analysis was performed to show the apoptotic cell percentage **(B)** and cycle distribution **(C)** in SHG-44 and U251 cells with or without ZNF655 knockdown. **(D, E)** Wound-healing assay **(D)** and Transwell assay **(E)** were performed to compare the cell migration ability of SHG-44 and U251 cells treated with shCtrl or shZNF655. The data were expressed as mean ± SD (n ≥ 3), **p < 0.01, ***p < 0.001.

### Knockdown of ZNF655 Attenuates Glioma Formation *In Vivo*

The effects of the downregulation of ZNF655 were further analyzed by the construction of the mouse xenograft model. The growth of mouse tumors was monitored for 65 days, and it was found that the tumor growth of the ZNF655 knockdown group was slower than that of the control group (p < 0.05) (**Figure 3A**). The *in vivo* imaging results on the 65th day showed that the fluorescence intensity of the shZNF655 group was weaker than that of shCtrl (p < 0.05), indicating that the downregulation of ZNF655 inhibited tumor formation in mice (**Figure 3B**). Subsequently, the tumors in the shZNF655 group were smaller in size and lighter in weight than those in shCtrl (p < 0.001), which could be more visually observed in the tumors removed from the mice (**Figure 3C**). Furthermore, the quantitative analysis of IHC in Ki67 indicated that the signal strength of the shZNF655 group was lower than that of shCtrl, reflecting that the knockdown of ZNF655 weakened the ability of tumor formation (**Figure 3D**). The above results together indicated that the downregulation of ZNF655 could attenuate tumor formation *in vivo*.

The article "ZNF655 Promotes the Progression of Glioma Through Transcriptional Regulation of AURKA" was retracted in 2023. Reasons: unreliable results or conclusions; concerns about the data.

**Figure 3:** Knockdown of ZNF655 inhibits tumor growth *in vivo*. **(A)** The growth of mouse tumors was monitored for 65 days and tumor volume in shCtrl and shZNF655 groups were measured. **(B)** The total fluorescent intensity of tumors in the shCtrl group and shZNF655 group was detected. **(C)** The xenograft tumors were removed from the model mice, and tumor weight was measured after the sacrifice of mouse models. **(D)** The Ki67 index of the removed tumors was evaluated by immunohistochemical staining analysis (×200 magnification and ×400 magnification). The data were expressed as mean ± SD (n ≥ 3), *p < 0.05, ***p < 0.001.

### ZNF655 Transcriptionally Regulates AURKA Expression

To further recognize the downstream targets of ZNF655 in regulation of glioma, we performed RNA sequencing analysis in U251 cells. The results of hierarchical clustering (**Figure 4A**) and volcano plot (**Figure S2A**) indicated that ZNF655 knockdown resulted in upregulation of 185 genes and downregulation of 514 genes in U251 cells. Further exploration based on IPA indicated that DEGs were mostly enriched in pathways related to cycle regulation (**Figure S2B**), especially affecting the cell cycle, growth, proliferation, movement, and other behaviors (**Figure S2C**). According to the selection criteria of DEGs, the top 5 genes enriched in these functions were selected through qPCR (**Figure S2D**) and WB (**Figure 4B**). AURKA has been shown to regulate the self-renewal and tumorigenicity of glioma-initiating cells (23), so we focused on AURKA.

**Figure 4:** ZNF655 directly binds to the AURKA promoter and regulates its activity. **(A)** Hierarchical clustering showed the DEGs of U251 cells after ZNF655 knockdown. **(B)** The expression of most significantly DEGs was identified by WB in U251 cells. **(C, D)** Effects of ZNF655 knockdown or overexpression on AURKA mRNA and protein expression. **(E)** We tested the effect of ZNF655 expression on AURKA promoter activity by constructing AURKA promotor dual luciferase reporter gene in U251 cells. **(F)** We performed ChIP-qPCR experiments to verify the mechanism of ZNF655 regulating AURKA. **(G)** The mRNA expression of AURKA was elevated in glioma cell lines (U87, U251, and SHG-44) and human brain normal glial cells HEB. **(H, I)** The expressions of AURKA in glioma tissue (n = 125; low grade, n = 49, high grade, n = 76) and normal tissue (n = 31) were analyzed through IHC staining (×200 magnification and ×400 magnification), and quantitative results of AURKA in gliomas were shown. **(J, K)** Based on the TCGA database, the expression levels of AURKA in glioblastoma and its correlation with survival were analyzed. The data were expressed as mean ± SD (n ≥ 3), **p < 0.01, ***p < 0.001.

The article "ZNF655 Promotes the Progression of Glioma Through Transcriptional Regulation of AURKA" was retracted in 2023. Reasons: unreliable results or conclusions; concerns about the data.

Subsequently, we found that the expression of AURKA was decreased in ZNF655 knockdown of U251 cells. Interestingly, the expression of AURKA was upregulated after ZNF655 overexpression (**Figures 4C, D**). These results suggested that ZNF655 may regulate the expression of AURKA in some way. On the other hand, as a member of ATF, ZNF655 could specifically transcriptionally regulate the expression of downstream target genes. Therefore, we inferred that ZNF655 transcriptionally regulated AURKA promoter activity. We tested the effect of ZNF655 expression on AURKA promoter activity by constructing the AURKA promotor dual luciferase reporter gene in U251 cells. Compared with the NC group, ZNF655 overexpression dramatically increased the AURKA promoter luciferase activity (**Figure 4E**). The results suggested that ZNF655 directly bound to the AURKA promoter and regulated its activity. In addition, we performed chromatin immunoprecipitation (ChIP)-qPCR experiments to verify the mechanism of ZNF655 regulating AURKA. Overexpression of ZNF655 increased antibody recovery in the upstream promoter region of AURKA, suggesting that binding of ZNF655 to the endogenous AURKA promoter region (**Figure 4F**). Thus, our findings clarified that ZNF655 could transcriptionally activate AURKA by directly interacting with the AURKA promoter.

### Knockdown of AURKA Reverses the Promoting Effects of ZNF655 Overexpression on Glioma Cells

Moreover, the mRNA expression of AURKA was elevated in glioma cell lines (U87, U251, and SHG-44) compared to human brain normal glial cells HEB (**Figure 4G**). AURKA expression in glioma was significantly higher than that in normal tissues (**Figure 4H**), as the quantitative results show in **Figure 4I**. As expected, the results based on the TCGA database further showed that the expression level of AURKA in glioblastoma (n = 155) was significantly higher than that of normal tissues (n =5) (**Figure 4J**). Although the survival time of glioblastoma with high AURKA expression was short, there was no significant correlation between them (**Figure 4K**). In addition, the effect of AURKA on glioma was evaluated in U251 cells using loss/gain of assays. ZNF655+shAURKA was the cell with downregulation of AURKA and overexpression of ZNF655 simultaneously. NC (KD+OE) was the BR-V-108 vector with control scrambled sequence for cell infection (**Figures S3A–I**). After AURKA downregulation, U251 cells showed decreased proliferation ability, enhanced apoptosis, and inhibited migration (**Figures S4A–D**). On the contrary, the overexpression of ZNF655 in U251 cells increased proliferation, decreased apoptosis, and promoted migration (**Figures 5A–E**). Compared with NC (KD+OE), the cells in the ZNF655+shAURKA group showed varying degrees of reduction in proliferation, apoptosis, and migration. Therefore, the recovery experiments verified that AURKA knockdown could alleviate the promoting effects of ZNF655 overexpression on glioma.

The article "ZNF655 Promotes the Progression of Glioma Through Transcriptional Regulation of AURKA" was retracted in 2023. Reasons: unreliable results or conclusions; concerns about the data.

**Figure 5:** AURKA knockdown alleviates the effects of ZNF655 overexpression on glioma cells. The effects of ZNF655 overexpression or AURKA knockdown on proliferation, apoptosis, cycle, and migration of U251 cells were examined by Celigo cell counting assay **(A)**, flow cytometry **(B, C)**, wound-healing assay **(D)**, and Transwell assay (×200 magnification) **(E)**, respectively. The data were expressed as mean ± SD (n ≥ 3), *p < 0.05, **p < 0.01, ***p < 0.001.

## Discussion

In this study, we found a significant positive correlation between the expression of ZNF655 and pathological data such as tumor grade as well as tumor recurrence. In addition, the expression of ZNF655 has important clinical significance in predicting the prognosis of glioma patients. Furthermore, knockdown of ZNF655 suppressed the progression of glioma cells, which was characterized by reduced proliferation, enhanced apoptosis, cycle repression in G2, inhibition of migration, and weakened tumorigenesis.

Previous studies have shown that decreased apoptosis is considered as an important factor in tumorigenesis and carcinogenesis (24). Subsequently, the study preliminarily investigated the effect of ZNF655 knockdown on the apoptosis signaling pathway in U251 cells by using human apoptotic antibody array. Interestingly, we found that knockdown of ZNF655 resulted in downregulation of Bcl-2, Bcl-w, clAP-2, IGF-I, IGF-II, sTNF-R1, sTNF-R2, and TNF-β. Tumor suppressors combine with pro-survival proteins of the Bcl-2 family such as Bcl-w and Bcl-XL to release Bax, which in turn exerts the functions of pro-apoptosis or anti-invasion (25). Anti-apoptotic factor clAP-2 maintains cell proliferation by regulating the dynamic stability of microtubules (26, 27). IGF-II differentially regulates IGF-I receptor signaling cascade and stimulates anti-apoptotic proteins Bcl-2 and Bcl-XL to prevent cell apoptosis (28). Moreover, tumor necrosis factor (TNF) and its soluble receptors type 1 (sTNF-R1) and type 2 (sTNF-R2) are considered to be key mediators of cancer cell apoptosis and progression (29). In this study, we found that ZNF655 knockdown would downregulate these anti-apoptotic proteins. However, the mechanism underlying the regulation of the apoptosis signaling pathway by ZNF655 remains to be further explored.

The article "ZNF655 Promotes the Progression of Glioma Through Transcriptional Regulation of AURKA" was retracted in 2023. Reasons: unreliable results or conclusions; concerns about the data.

According to results of RNA sequencing, AURKA was preliminarily identified as a downstream target of ZNF655 involved in glioma regulation in this study. AURKA is a serine–threonine kinase, located on chromosome 20q, which exerts roles in mitotic spindle formation and chromosome segregation (30, 31). The abnormality of AURKA leads to mitotic spindle assembly checkpoint coverage; polyploid cells produce excessive centrosomes and genetic instability (32–34). An abnormally high expression of AURKA has been identified in breast, lung, ovarian, colorectal, gastric, and esophageal cancers (35–41). Overexpression of AURKA has carcinogenic characteristics (42). Studies have shown that AURKA promotes tumor development by regulating cell proliferation, migration, invasion, epithelial mesenchymal transition, and cancer stem cell behavior (43–45). Inhibition of AURKA activity can reduce the proliferation and survival of gastrointestinal cancer cells (46). Several small molecular inhibitors of AURKA have shown therapeutic effects in preclinical studies (47, 48). Additionally, Willems et al. illuminated that AURKA contributed to the survival, proliferation, radiation resistance, and self-renewal of glioblastoma cells (49). Obviously, AURKA played a crucial role in the regulation of tumor growth, which may be an extremely valuable therapeutic target. Of note, the present study further revealed that ZNF655 could transcriptionally activate AURKA by directly interacting with the AURKA promoter. Additionally, knockdown of AURKA reversed the promoting effects of ZNF655 overexpression on glioma cells.

This study illustrated the promoting effect of ZNF655 on glioma. High expression of ZNF655 contributed to the deterioration of glioma by binding to the promoter of AURKA and was associated with a poor prognosis. Therefore, ZNF655 may be a promising target for molecular therapy of glioma.

## Data Availability Statement

The original contributions presented in the study are included in the article/**Supplementary Material**. Further inquiries can be directed to the corresponding author.

## Ethics Statement

This study was approved by the Research Ethics Committee of the First Affiliated Hospital of Zhengzhou University. The patients/participants provided their written informed consent to participate in this study. All procedures involving mice and experimental protocols were approved by the Institutional Animal Care and Use Committees of the Neurosurgery, Tongji Hospital, Tongji Medical College, Huazhong University of Science and Technology.

The article "ZNF655 Promotes the Progression of Glioma Through Transcriptional Regulation of AURKA" was retracted in 2023. Reasons: unreliable results or conclusions; concerns about the data.

## Author Contributions

PZ designed this program. ZZ, CL, MW, and HS operated the cell experiments. XC performed the animal experiments. All authors contributed to the article and approved the submitted version.

## Conflict of Interest

The authors declare that the research was conducted in the absence of any commercial or financial relationships that could be construed as a potential conflict of interest.

## Publisher’s Note

All claims expressed in this article are solely those of the authors and do not necessarily represent those of their affiliated organizations, or those of the publisher, the editors and the reviewers. Any product that may be evaluated in this article, or claim that may be made by its manufacturer, is not guaranteed or endorsed by the publisher.
